# Diagnostic value of high‐frequency ultrasound (HFUS) in evaluation of subcutaneous lesions

**DOI:** 10.1111/srt.13464

**Published:** 2023-09-10

**Authors:** Yao Miao, Wei‐Wei Ren, Fei‐Yue Yang, Liang Li, Ling Wu, Dan‐ Dan Shan, Zi‐Tong Chen, Li‐Fan Wang, Qiao Wang, Le‐Hang Guo

**Affiliations:** ^1^ Department of Medical Ultrasound Shanghai Tenth People's Hospital; Shanghai Engineering Research Center of Ultrasound Diagnosis and Treatment School of Medicine Tongji University Shanghai China; ^2^ Department of Medical Ultrasound Shanghai Skin Disease Hospital School of Medicine Tongji University Shanghai China; ^3^ Department of Dermatological Surgery Shanghai Skin Disease Hospital School of Medicine Tongji University Shanghai China; ^4^ Department of Ultrasound Zhongshan Hospital Fudan University Shanghai China

**Keywords:** dermatology, subcutaneous lesions, ultrasound

## Abstract

**Background:**

It is unknown whether high‐frequency ultrasound (HFUS) can evaluate invisible subcutaneous lesions. We aimed to investigate the diagnostic value of HFUS in invisible subcutaneous lesions.

**Method:**

Patients with invisible subcutaneous lesions were prospectively recruited from two centres. Before undergoing biopsy or surgery, each lesion was independently evaluated by two clinicians. One provides a clinical diagnosis by only clinical examination and the other provides an integrated diagnosis by combining clinical examination and HFUS information. Diagnoses were classified as correct, wrong, and indeterminate. A total of 391 lesions from 355 patients were enrolled, including 225 epidermoid cysts, 77 lipomas, 25 pilomatrixomas, 21 haemangiomas, 19 dermatofibromas, 11 dermatofibrosarcoma protuberans (DFSP), 7 neurofibromas, and 6 leiomyomas. Using pathological results as the gold standard, diagnostic performance was compared.

**Results:**

The number of correct diagnoses increased from 185 (47.3%) by clinical examination alone to 316 (80.8%) after the addition of HFUS (P < 0.05). Meanwhile, the indeterminate diagnosis rate decreased from 143 (36.6%) to 10 (2.6%). Using HFUS, the accuracy improved significantly for epidermoid cysts (59.6% vs. 86.7%), lipomas (50.6% vs. 94.8%), pilomatrixomas (0% vs. 48.0%), haemangiomas (23.8% vs. 57.1%), and DFSPs (0% vs. 81.8%) (all *p* < 0.05). However, HFUS did not significantly improve the diagnostic accuracy of dermatofibromas (15.8% vs. 21.1%, *p* > 0.999), neurofibromas (42.9% vs. 71.4%, *p* = 0.625), or leiomyomas (16.7% vs. 100%, *p* = 0.063).

**Conclusion:**

Combining HFUS and clinical examination can generally improve the diagnostic accuracy and decrease the indeterminacy of invisible subcutaneous lesions, especially epidermoid cysts, lipomas, pilomatrixomas, haemangiomas, and DFSPs. However, for some rare lesions, HFUS cannot provide useful information.

## 1 INTRODUCTION

Lesions located in the subcutaneous tissue are very common, with an incidence of approximately 3 per 1000 people per year. When dealing with these lesions, the first question dermatologists have is whether the lesions could be malignant. However, most are only palpable but invisible.^1^, ^2^, ^3^, ^4^ Thus, dermatologists must evaluate underlying lesions using non‐visual information such as medical history and physical examination. Therefore, the diagnosis of subcutaneous lesions is difficult due to nonspecific presentation, and many patients may receive an incorrect action plan, such as unnecessary biopsy or delayed treatment.^5^, ^6^ In this setting, imaging can be used to provide a provisional or definitive diagnosis of the underlying lesions.^7^

Several imaging modalities have been used to assess subcutaneous lesions. According to the American College of Radiology Appropriateness Criteria about Soft‐Tissue Masses, computed tomography (CT) is usually not appropriate because of radiation exposure and limited definition.^8^ Magnetic resonance imaging (MRI) at 3T with appropriate surface coil has perfect skin resolution.^9^ And MRI could provide perfect correlation between lesion depth and histology.^10^ With appropriate techniques, MRI now provides almost microscopic type of analysis to achieve visualization of hair follicles.^11^ However, MRI is significantly expensive, time‐consuming, and not readily available.^8^, ^9^ On the other hand, dermatoscopy, optical coherence tomography (OCT), and reflectance confocal microscopy (RCM) have limited penetration, all of which are incapable of diagnosing lesions located in subcutaneous soft tissues.^12^

Compared with the above‐mentioned modalities, ultrasound (US) is balanced for resolution and penetration, so it has the potential to evaluate underlying lesions located in subcutaneous tissue.^13^, ^14^, ^15^, ^16^, ^17^, ^18^, ^19^, ^20^ With the development of high‐frequency ultrasound (HFUS), the resolution is continuously improving, thus dermatological lesions can be well evaluated.^21^, ^22^, ^23^ In evaluation of skin subcutaneous lesions, HFUS is now used for image guided superficial radiation therapy and Doppler modality is starting to be utilized in evaluation of vasculature of all skin lesions.^24^, ^25^, ^26^

It should be noted that, so far as we know, most of the previous studies regarding the usefulness of HFUS were with a visible change of appearance. The appearance of lesions can provide additional diagnostic information. However, the clinical benefits of HFUS have not been confirmed for invisible lesions located in subcutaneous tissue.

Therefore, since lesions in the dermatology department are usually small and superficial, we hypothesise that combining HFUS might provide more useful information for dermatologists so that they can better understand these invisible subcutaneous lesions.

## 2 MATERIALS AND METHODS

The study protocol was approved by the hospital ethics committee. All patients were informed and agreed to use their data for this study.

### 2.1 Study design

This prospective study followed the principles of the Declaration of Helsinki. This study protocol was reviewed and approved by the Institutional Review Board and the Ethics Committee (Approval number: SHSY‐IEC‐5.0/22K297/P01). The primary purpose of the study was to investigate whether HFUS can add benefits to clinical practice in general. The secondary purpose was to investigate the performance of HFUS in the diagnosis of a specific type of lesion. The study was registered at https://www.chictr.org.cn (No. ChiCTR2300068635).

### 2.2 Data acquisition

From December 2016 to July 2021, the prospective study was conducted at Shanghai Tenth People's Hospital and Shanghai Skin Disease Hospital. Patients with invisible subcutaneous lesions who visited the dermatology department were recruited. The invisible subcutaneous lesion was defined as a palpable or protrusion‐like lesion, but without any significant pigmentation, sinus tract, ulceration, or redness.

The inclusion criteria were as follows: (a) the patient underwent HFUS examination; (b) a pathological result for each lesion was available after biopsy or surgery. Patients who fulfilled one of the following criteria were excluded: (a) the lesion had a treatment history before the HFUS examination; (b) the pathological result was indefinite; (c) umbilical and inguinal hernias, lesions located deep in the muscular layer, or lesions of organic origin such as thyroid or breast (Figures 1 and 2).

**FIGURE 1:** Images obtained from a 63‐year‐old male patient with epidermoid cyst (A and B). (A) The lesion was invisible to the naked eye but could be palpated (arrows). (B) The grayscale image of epidermoid cyst (arrows) shows that the lesion is homogeneous with posterior acoustic enhancement.

**FIGURE 2:** Process of patient enrollment in the study.

Clinicians were divided into roles A (*n* = 10) and B (*n* = 3). The clinical experience of the two roles was comparable; however, the roles B could perform HFUS skilfully (with 3−7 years of experience in skin HFUS).

### 2.3 Patients’ characteristics

In total, 446 patients were recruited for this study. Among them, 73 patients with a treatment history before the HFUS examination, 11 patients with indefinite pathological results, 3 patients with umbilical hernias, and 4 patients with inguinal hernias were excluded. Ultimately, 355 patients (219 males and 136 females) aged 5 to 86 years (mean age, 47.6 ± 17.8 years) were enrolled, of which 27 patients had more than two lesions. Of the 391 lesions, 380 were benign and 11 malignant. There were epidermoid cysts (57.5%, 225/391), lipomas (19.7%, 77/391), pilomatrixomas (6.4%,25/391), haemangiomas (5.4%, 21/319), dermatofibromas (4.9%, 19/391), DFSPs (2.8%, 11/391), neurofibromas (1.8%, 7/391), and leiomyomas (1.5%, 6/391) (Table 1).

**TABLE 1:** Baseline characteristics of patient and disease.

Characteristics	*N*
No. of patients	355
Patient sex	
No. of men	219
No. of women	136
Mean age (years)	47.6 ± 17.8
No. of subcutaneous masses	391
Epidermoid cyst	225 (57.5%)
Lipoma	77 (19.7%)
Pilomatrixoma	25 (6.4%)
Haemangioma	21 (5.4%)
Dermatofibroma	19 (4.9%)
DFSP	11 (2.8%)
Neurofibroma	7 (1.8%)
Leiomyoma	6 (1.5%)

Data for mean age are mean ± standard deviation. Data in parentheses are percentages.

DFSP, dermatofibrosarcoma protuberans.

### 2.4 Clinical diagnoses

After referring to the ultrasound consensus,^20^ the clinical diagnosis of each invisible subcutaneous lesion was independently provided by a clinician of role A by clinical examination through palpation, medical history, and the patient's symptoms. Subsequently, the participant was referred to another clinician of role B for further evaluation. The diagnosis of role A for each lesion was blinded to that of role B.

### 2.5 Combined diagnosis of HFUS and clinical examination

For the same participant, in addition to clinical features through palpation, medical history, and the patient's symptoms, a clinician of role B additionally performed the HFUS examination using a MyLab TMC class scanner (Esaote SpA; Genoa, Italy) with a linear transducer (frequency range, 6−18 MHz) or SuperSonic Imagine with the Aixplorer US system with a linear transducer (frequency range, 10−22 MHz). When some lesions were found to be invisible or unclear in the HFUS examination, they were evaluated in detail with Ultra‐high frequency ultrasound imaging system‐Paragon XHD (22−38 MHz, KOLO, Jiangsu, China).

Patients were asked to select an appropriate examination position to fully expose the lesion. HFUS parameters, such as frequency, gain, depth, and focus, were adjusted to ensure clarity for each lesion. Multisection scanning was performed for each lesion to measure the maximum diameter. Colour Doppler flow imaging (CDFI) was performed. Similarly, after referring to the ultrasound consensus,^20^ clinicians make the final diagnosis after combining clinical experience with relevant guidelines by observing the imaging features such as morphology, echogenicity, layer involvement and CDFI signal, and so on.

### 2.6 Diagnosis

The clinical diagnosis and combined diagnosis of HFUS and clinical examination were both classified as three conditions: correct diagnosis, wrong diagnosis, and indeterminate diagnosis. Pathological results were the gold standard. Classification of correct and wrong diagnoses was based on pathological results. An indeterminate diagnosis included no clinical diagnoses or uncertain clinical diagnoses.

### 2.7 Statistical analysis

Statistical analysis was performed using Statistical Package for the Social Sciences version 26.0 (IBM, Armonk, New York, USA) software. The chi‐squared test and McNemar test were used to analyse differences between the diagnostic accuracy of integrated diagnosis and clinical diagnosis, with pathological results as the gold standard. A *p* value less than 0.05 was considered statistically significant.

## 3 RESULTS

### 3.1 Clinical benefits of HFUS in general

As shown in Tables 2 and 3, of the 391 lesions, 185 lesions (47.3%) were correctly diagnosed by clinical examination, 63 lesions (16.1%) were misdiagnosed, and 143 lesions (36.6%) were indeterminately diagnosed in clinical examination. The overall accuracy of clinical diagnosis was 47.3% (185/391). When taking six relatively rare diseases, including pilomatrixoma, haemangioma, DFSP, dermatofibroma, neurofibroma, and leiomyoma as a whole, the diagnostic accuracy of clinical diagnosis was only 13.5% (12/89).

**TABLE 2:** Comparison of clinical diagnosis and combined diagnosis.

Diseases	Correct clinical diagnosis	Correct combined diagnosis	*p*
Epidermoid cyst	59.6% (134/225)	86.7% (195/225)	<0.001^*^
Lipoma	50.6% (39/77)	94.8% (73/77)	<0.001^*^
Pilomatrixoma	0 (0/25)	48.0% (12/25)	<0.001^*^
Haemangioma	23.8% (5/21)	57.1% (12/21)	0.021^*^
DFSP	0 (0/11)	81.8% (9/11)	0.004^*^
Dermatofibroma	15.8% (3/19)	21.1% (4/19)	>0.999
Neurofibroma	42.9% (3/7)	71.4% (5/7)	0.625
Leiomyoma	16.7% (1/6)	100.0% (6/6)	0.063
The last six diseases^a^	13.5% (12/89)	53.9% (48/89)	<0.001^*^
Total	47.3% (185/391)	80.8% (316/391)	<0.001^*^

Data in parentheses are the number of correctly diagnosed cases divided by the total number.

DFSP, dermatofibrosarcoma protuberans.

^a^ Refers to the sum of pilomatrixoma, haemangioma, DFSP, dermatofibroma, neurofibroma and leiomyoma (*n* = 89).

* Statistically significant difference between the two groups (*p* < 0.05).

**TABLE 3:** Comparison of clinical diagnosis and combined diagnosis.

Diseases	Wrong clinical diagnosis	Wrong combined diagnosis	*p*	Indeterminate clinical diagnosis	Indeterminate combined diagnosis	*p*
Epidermoid cyst	8.9% (20/225)	12.0% (27/225)	0.307	31.5% (71/225)	1.3% (3/225)	<0.001^*^
Lipoma	13.0% (10/77)	3.9% (3/77)	0.052	36.4% (28/77)	1.3% (1/77)	<0.001^*^
Pilomatrixoma	60.0% (15/25)	48.0% (12/25)	0.563	40.0% (10/25)	4.0% (1/25)	0.006^*^
Haemangioma	38.1% (8/21)	28.6% (6/21)	0.593	38.1% (8/21)	14.3% (3/21)	0.132
DFSP	27.3% (3/11)	9.1% (1/11)	0.317	72.7% (8/11)	9.1% (1/11)	0.020^*^
Dermatofibroma	26.3% (5/19)	78.9% (15/19)	0.025^*^	57.9% (11/19)	0 (0/19)	<0.001^*^
Neurofibroma	14.2% (1/7)	14.2% (1/7)	1.000	42.9% (3/7)	14.2% (1/7)	0.317
Leiomyoma	16.7% (1/6)	0 (0/6)	0.317	66.7% (4/6)	0 (0/6)	0.046^*^
Total	16.1% (63/391)	16.6% (65/391)	0.860	36.6% (143/391)	2.6% (10/391)	<0.001^*^

Data in parentheses are the number of wrong or indeterminate diagnosed cases divided by the total number.

DFSP , dermatofibrosarcoma protuberans.

* Statistically significant difference between the two groups (*p* < 0.05).

After adding HFUS, the combined diagnosis achieved higher accuracy overall (80.8% vs. 47.3%, *p* < 0.05). When we combined the six rare diseases in our study, the combined diagnosis of HFUS and clinical features significantly improved from 13.5% (12/89) to 53.9% (48/89) (*p* < 0.05).

### 3.2 The performance of HFUS in diagnosing a specific kind of lesion

As shown in Tables 2 and 3, the accuracy of clinical diagnosis for epidermoid cysts and lipomas was higher than the overall accuracy, with 59.6% (134/225) and 50.6% (39/77) versus 47.3% (185/391) (*p* = 0.042 and *p* = 0.699), respectively. However, the diagnostic accuracy of the six rare diseases was below the entirety, including pilomatrixoma (0/25), haemangioma (5/21), DFSP (0/11), dermatofibroma (3/19), neurofibroma (3/7), and leiomyoma (1/6), ranging from 0% to 42.9%.

Compared with clinical diagnosis, after adding HFUS, the accuracy improved significantly for epidermoid cysts (59.6% vs. 86.7%), lipomas (50.6% vs. 94.8%), pilomatrixomas (0% vs. 48.0%), haemangiomas (23.8% vs. 57.1%), and DFSPs (0% vs. 81.8%) (all *p* < 0.05). Meanwhile, although the accuracy improved, there was no significant difference between the clinical diagnosis and combined diagnosis of dermatofibroma (15.8% vs. 21.1%, *p* > 0.999), neurofibroma (42.9% vs. 71.4%, *p* = 0.625), or leiomyoma (16.7% vs. 100%, *p* = 0.063) (Table 2 and Figure 3).

**FIGURE 3:** Correct clinical diagnosis and combined diagnosis.

As shown in Table 4, the performance of the combined diagnosis of HFUS and clinical settings in different clinical diagnostic situations was analysed. First, among the lesions with a correct clinical diagnosis, the accuracy of the HFUS diagnosis was 90.3% (167/185). Eighteen (10.8%) lesions were incorrectly or indeterminately diagnosed by HFUS, including 13 epidermoid cysts, 2 haemangiomas, 2 dermatofibromas, and 1 neurofibroma.

**TABLE 4:** The ability of combined diagnosis.

	Correct clinical diagnosis(*n* = 185)		Wrong clinical diagnosis(*n* = 63)		Indeterminate clinical diagnosis(*n* = 143)	
Diseases	Correct combined diagnosis	Wrong or indeterminate combined diagnosis	Correct combined diagnosis	Wrong or indeterminate combined diagnosis	Correct combined diagnosis	Wrong or combined diagnosis
Epidermoid cyst	90.3% (121/134)	9.7% (13/134)	75.0% (15/20)	25.0% (5/20)	83.1% (59/71)	16.9% (12/71)
Lipoma	100.0% (39/39)	0 (0/39)	90.0% (9/10)	10.0% (1/10)	89.3% (25/28)	10.7% (3/28)
Pilomatrixoma	0	0	53.3% (8/15)	46.7% (7/15)	40.0% (4/10)	60.0% (6/10)
Haemangioma	60.0% (3/5)	40.0% (2/5)	62.5% (5/8)	37.5% (3/8)	50.0% (4/8)	50.0% (4/8)
DFSP	0	0	66.7% (2/3)	33.3% (1/3)	87.5% (7/8)	12.5% (1/8)
Dermatofibroma	33.3% (1/3)	66.7% (2/3)	20.0% (1/5)	80.0% (4/5)	18.2% (2/11)	81.8% (9/11)
Neurofibroma	66.7% (2/3)	33.3% (1/3)	0 (0/1)	100.0% (1/1)	100.0% (3/3)	0 (0/3)
Leiomyoma	100.0% (1/1)	0 (0/1)	100.0% (1/1)	0 (0/1)	100.0% (4/4)	0 (0/4)
Total	90.3% (167/185)	9.7% (18/185)	65.1% (41/63)	34.9% (22/63)	75.5% (108/143)	24.5% (35/143)
The last six diseases^a^	75.0% (9/12)	25.0% (3/12)	51.5% (17/33)	48.5% (16/33)	54.5% (24/44)	45.5% (20/44)

Data in parentheses are the number of correct or wrong or indeterminate diagnosed cases divided by the total number.

DFSP , dermatofibrosarcoma protuberans.

^a^ Refers to the sum of pilomatrixoma, haemangioma, dermatofibrosarcoma protuberan, dermatofibroma, neurofibroma, and leiomyoma.

Second, in the clinical diagnosis, 60 benign lesions and 3 malignant lesions were misdiagnosed. Of these, 41 lesions were corrected by adding HFUS with an accuracy of 65.1% (41/63), including 75.0% (15/20) epidermoid cysts, 90.0% (9/10) lipomas, 53.3% (8/15) pilomatrixomas, 62.5% (5/8) haemangiomas, 66.7% (2/3) DFSPs, 20.0% (1/5) dermatofibromas, and 100% (1/1) leiomyomas. Among the lesions that were clinically misdiagnosed, although 22 lesions were incorrectly diagnosed by HFUS, 21 lesions, including five epidermoid cysts, one lipoma, seven pilomatrixomas, three haemangiomas, four dermatofibromas, and one neurofibroma, were diagnosed as other benign entities, and only one DFSP was indeterminately diagnosed.

Finally, 143 lesions had an indeterminate clinical diagnosis. Among these lesions, HFUS correctly diagnosed 108 lesions with an accuracy of 75.5% (108/143). HFUS correctly diagnosed 83.1% (59/71) of epidermoid cysts, 89.3% (25/28) of lipomas, 40.0% (4/10) of pilomatrixomas, 50.0% (4/8) of haemangiomas, 87.5% (7/8) of DFSPs, 18.2% (2/11) of dermatofibromas, 100% (3/3) of neurofibromas, and 100% (4/4) of leiomyomas. However, 24.5% (35/143) of lesions were not correctly diagnosed by HFUS, including 12 epidermoid cysts, three lipomas, six pilomatrixomas, four haemangiomas, one DFSP and nine dermatofibromas. Therefore, further examinations are needed to confirm the diagnoses (Figures 4 and 5).

**FIGURE 4:** Comparison of clinical diagnosis (C D) and combined clinical examination and HFUS information diagnosis (U+C D). (A) Epidermoid cyst. (B) Lipoma. (C) Haemangioma. (D) Pilomatrixoma. (E) Dermatofibrosarcoma protuberans (DFSP). (F) All lesions.

**FIGURE 5:** Comparison of clinical diagnosis (C D) and combined clinical examination and HFUS information diagnosis (U+C D). Data in parentheses are percentages. (A) Dermatofibroma. (B) Neurofibroma. (C) Leiomyoma. (D) The last six diseases, including pilomatrixoma, haemangioma, DFSP, dermatofibroma, neurofibroma and leiomyoma.

## 4 DISCUSSION

In the present study, we analysed the value of HFUS in the diagnosis of invisible subcutaneous lesions. The results demonstrated that HFUS was valuable and showed a higher accuracy than that based on clinical diagnosis alone. This result could be helpful for accurately diagnosing most benign lesions and decreasing the number of indeterminate lesions.

Wortsman et al. performed a retrospective study of 4468 skin lesions, including visible and invisible lesions, and compared US diagnosis with clinical diagnosis. The diagnostic accuracy of the referred diagnosis was 73%, and the addition of ultrasound increased the accuracy to 97%. We noticed that the diagnostic accuracy of HFUS was higher than that in the present study.^27^ The reason for this might be that most of the skin lesions they studied were visible to the naked eye. With visualised information, diagnostic accuracy can be improved. However, the diagnostic accuracy of HFUS for invisible subcutaneous lesions has not been studied extensively. Hwang et al. retrospectively characterised the subcutaneous lesions. The results showed that the accuracy was 52.0% for clinical diagnosis and 82.0% for US,^16^ which is consistent with the present study. However, only benign lesions were included in the study. Both benign and malignant lesions were enrolled in our study, therefore, our design may be closer to clinical practice.

In the present study, the most common entity was epidermoid cysts, which is consistent with previous studies.^16^, ^17^ However, other studies have suggested that lipomas are the most common. This may be related to the different regions and experimental methods.^28^, ^29^

Traditionally, diagnosis of the two most common lesions has not been considered a critical issue. However, nearly half of these lesions were indeterminate. Therefore, these patients may undergo unnecessary biopsies or treatment. Fortunately, our study showed that HFUS significantly improved the diagnostic accuracy for lipomas from 50.6% to 94.8% and for epidermoid cysts from 59.6% to 85.8%, compared with clinical diagnosis alone. Similarly, Kuwano et al. found that HFUS increased the diagnostic accuracy for lipomas from 54.8% to 88.1% and the diagnostic accuracy for epidermoid cysts from 43.2% to 65.9%, compared with palpation alone by the clinician.^17^ Therefore, HFUS may help to avoid overtreatment.

However, some common lesions are not accurately diagnosed by HFUS. We also found that 12.0% (27/225) of epidermoid cyst lesions had not been correctly diagnosed but were misdiagnosed as other entities, such as inflammatory lesions, trichilemmal cysts, and lipomas, due to their similar internal echoes or secondary changes. For example, when an epidermoid cyst ruptures, the contents inside are lost. Therefore, the lesion might change its original oval shape to an irregular shape, and the echogenicity of the lesion is heterogeneous. Moreover, the soft tissue around the lesion usually swells. Therefore, the lesion may easily be misdiagnosed as a subcutaneous malignancy. Likewise, when some epidermoid cysts had prolonged accumulation of blood and necrotic keratin debris, the performance in HFUS was similar to that of some trichilemmal cysts with foci of calcification (Tables 3 and 4).

In contrast, the performance of HFUS for lipomas was relatively stable, and it correctly diagnosed more lesions in our study. In only 3.9% (3/77) of the lesions, HFUS failed to provide a correct diagnosis, and they were diagnosed with calcification and indeterminate lesions. This may be related to unrepresentative HFUS characteristics.

Statistically, for some relatively rare lesions, including pilomatrixoma, haemangioma, and DFSP, combined diagnosis is generally superior to clinical diagnosis in the present study. However, for certain specific lesions, the performance is unsatisfactory in real practice. In the pilomatrixoma group, only 48.0% (12/25) of the lesions were correctly diagnosed. Common mistakes included epidermoid cysts, lipomas, trichilemmal cysts, and inflammatory lesions. Similarly, the diagnostic accuracy for haemangiomas was 57.1% (12/21). The misdiagnosis was usually an epidermoid cyst or lipoma. This may be caused by the variety and complexity of HFUS manifestations in the relatively rare lesions in this study. In addition, a lack of experience may influence diagnosis accuracy.

DFSP was the only malignant lesion that was identified in this study. On the one hand, 81.8% (9/11) of the lesions were diagnosed correctly with the typical manifestations of HFUS, but on the other hand, 18.2% (2/11) of the lesions were still misdiagnosed because of the influence of inflammatory changes around the lesions or the influence of internal haemorrhage and necrosis of the lesions.

Based on our results, HFUS is currently unable to accurately diagnose dermatofibromas, neurofibromas, and leiomyomas. HFUS cannot correctly diagnose these lesions for the following reasons: First, their HFUS specificity may not be significant enough to identify them. Second, these three diseases were all relatively rare in our study, and the small number of lesions in practice may not provide sufficient experience for dermatologists. Therefore, we do not recommend that dermatologists diagnose invisible subcutaneous lesions as dermatofibromas, neurofibromas, or leiomyomas.

The limitations of this study are as follows: First, we only included invisible subcutaneous lesions with pathological results, which may lead to sampling bias, because most subcutaneous lesions, especially those considered benign, may not undergo biopsy or surgery under real conditions, so they were excluded without pathological results. Second, some subcutaneous pseudo‐tumours, such as hernias and cryptorchidism, were not included in the study. Meanwhile, some nodules in glands, including a large thyroid, parotid mixed tumour, and parotid Warthin tumour, were also not included in our study because they were not in the subcutaneous soft tissue. In addition, some umbilical and inguinal hernias were excluded from this study because the diagnosis of these diseases depends more on the intraoperative judgment of clinicians than on the pathological gold standard. However, they cannot be ignored in clinical practice. The performance of HFUS to diagnose these lesions mentioned needs to be further investigated. Third, the malignant lesions were relatively few in the study, thus, the efficiency of HFUS in differentiating between benign and malignant subcutaneous lesions has not been fully evaluated.

In conclusion, compared to clinical diagnosis, the combined diagnosis of HFUS and clinical examination can generally improve the diagnosis accuracy and decrease the number of unconfirmed cases of invisible subcutaneous lesions. In detail, combined diagnosis can correctly diagnose more epidermoid cysts, lipomas, pilomatrixomas, haemangiomas, and DFSPs compared to clinical diagnoses. However, for some relatively rare cases in our study, such as dermatofibromas, neurofibromas, and leiomyomas, HFUS failed to provide useful information.

## Data Availability

The data related to patients are not available for public access due to patient privacy requirements but can be obtained from the corresponding author on reasonable request after being approved by the institutional review board.
